RETRACTED

# Genome assembly of *M. spongiola* and comparative genomics of the genus *Morchella* provide initial insights into taxonomy and adaptive evolution

**DOI:** 10.1186/s12864-024-10418-8

**Published:** 2024-05-27

**Authors:** Qing Meng, Zhanling Xie, Hongyan Xu, Jing Guo, Qingqing Peng, Yanyan Li, Jiabao Yang, Deyu Dong, Taizhen Gao, Fan Zhang

**Affiliations:** 1 Qinghai University, 251 Ningda Road, Xining, Qinghai 810016 China; 2 Qinghai University of Technology, 15 Twenty-fourth Road, Xining, Qinghai 810016 China; 3 State-owned forest farms of Tianjun County, Delingha, Qinghai 817299 China; 4 Forestry and grassland station of Tianjun County, Delingha, Qinghai 817299 China

**Keywords:** *Morchella spongiola*, Genome assembly, Comparative genome, Evolution, Qinghai-Tibet Plateau

## Abstract

*Morchella spongiola* is a highly prized mushroom for its delicious flavor and medical value and is one of the most flourishing, representative, and dominant macrofungi in the Qilian Mountains of the Qinghai-Tibet Plateau subkingdoms (QTPs). However, the understanding of *M. spongiola* remains largely unknown, and its taxonomy is ambiguous. In this study, we redescribed a unique species of *M. spongiola*, i.e., micromorphology, molecular data, genomics, and comparative genomics, and the historical biogeography of *M. spongiola* were estimated for 182 single-copy homologous genes. A high-quality chromosome-level reference genome of *M. spongiola* M12-10 was obtained by combining PacBio HiFi data and Illumina sequencing technologies; it was approximately 57.1 Mb (contig N50 of 18.14 Mb) and contained 9775 protein-coding genes. Comparative genome analysis revealed considerable conservation and unique characteristics between *M. spongiola* M12-10 and 32 other *Morchella* species. Molecular phylogenetic analysis indicated that *M. spongiola* M12-10 is similar to the *M. prava*/*Mes*-7 present in sandy soil near rivers, differentiating from black morels ~ 43.06 Mya (million years ago), and diverged from *M. parva*/*Mes*-7 at approximately 12.85 Mya (in the Miocene epoch), which is closely related to the geological activities in the QTPs (in the Neogene). Therefore, *M. spongiola* is a unique species rather than a synonym of *M. vulgaris*/*Mes*-5, which has a distinctive grey-brown sponge-like ascomata. This genome of *M. spongiola* M12-10 is the first published genome sequence of the species in the genus *Morchella* from the QTPs, which could aid future studies on functional gene identification, germplasm resource management, and molecular breeding efforts, as well as evolutionary studies on the *Morchella* taxon in the QTPs.

**Supplementary Information:**

The online version contains supplementary material available at 10.1186/s12864-024-10418-8.

RETRACTED

## Introduction

Species of *Morchella* Dill. ex Pers. (Ascomycota, Pezizomycetes) are highly sought-after and prized edible fungi. They are not only delicious in flavor but also contain a biologically active substance that regulates immunity, anti-fatigue, antioxidant, antibacterial, antitumor [1–3], etc. Popular research aims have included taxonomy, medicinal efficacy, artificial cultivation, evolution of sexual reproduction, changes in chromosome ploidy, mating systems, transformation of reproductive type, development of zygotes, species evolution, and the historical biogeography of *Morchella* species [4–9]. Over 80 species-level lineages of *Morchella* have been inferred using molecular phylogenetics in recent years; the distribution of *Morchella* exhibits a high level of cryptic speciation and provincialism due to phenotypic plasticity and unreliable morphological species recognition [10–12]. Therefore, some of *Morchella*’s early described species appear to correspond to a variety of taxonomic systems. As with other famous *Morchella* species, *Morchella spongiola* Boud. has important ecological functions and high commercial value around the world and its distribution is restricted to temperate latitudes in the Northern Hemisphere, including Armenia, the Czech Republic, Denmark, Estonia, France, Germany, India, Norway, Pakistan, Slovakia, China, and Ukraine [6, 12, 13]. Meanwhile, *M. spongiola* is a well-known local wild economic product that is widely distributed in the Qilian Mountains of the Qinghai-Tibet Plateau subkingdoms (QTPs), where it grows abundantly on sandy soils, buckthorn woods near rivers, *Populus przewalskii Maxim.* forestry [14], ect. However, the taxonomy of *M. spongiola* is controversial because of the lack of complete morphological, molecular, and genomic data.

Among the thousands of species recorded in the fungal genome project, the genome project of *Morchella* first started in 2014. The genomes of *M. importuna*/*Mel*-10, *M. sextelata*/*Mel*-6, *M. septimelata*, and *M. crassipes* have already been published, and the JGI database also contains genomic records of 35 phylogenetic *Morchella* species [13]. The genomic sequencing of phylogenetic *Morchella* species has been helpful for specific genetic, phylogenetic, metabolic, and evolution studies [15–19]. Additionally, genome sequencing analysis promotes a further understanding of the polarity, taxonomy, life cycles, and nutritional ecotypes of fungi, such as *Tuber melanosporum* [20], *Laccaria bicolor* [21], *Stropharia rugosoannulata* [22], *Floccularia luteovirens* [23], and *Morchella crassipes* [24]. However, the inability to record a whole living history under laboratory conditions in earlier periods led to the stagnation of many biological studies on the *Morchella* species; these genomic studies were delayed more than those of other species. The genome of *Morchella spongiola* has not yet been published, which has hampered wide comparative genomic analysis across different fungal species. Here, we report a draft genome sequence of *M. spongiola* strain M12-10 using single molecule real-time (SMRT) sequencing. We then annotated the genome, conducted a comparative genomic analysis, and redescribed the taxonomy of *M. spongiola* based on morphological, molecular biological, genomic, and comparative genomic analyses. This valuable genomic resource will aid future studies on the evolution of *M. spongiola* and the genus *Morchella*, as well as studies on its evolutionary history.

RETRACTED

## Materials and methods

### Sampling information

Wild *Morchella* were collected from the Baokou River in the Qilian Mountains located on the QTPs annually in early May, with the GPS coordinates exhibited in Fig. 1A. The ascocarps of each collection were photographed in situ, and the altitude, surrounding vegetation, and substrate composition were documented. Dr. Xie Zhanling and Dr. Xu Hongyan undertook the formal identification of the plant material, and the identification of the plant material follows https://www.cfh.ac.cn/. Voucher specimens were deposited in Extreme Environment Microbiology Laboratory, Qinghai University, Xining, China.

**Fig. 1:** Information on *M. spongiola* M12-10. (**A**) Schematic diagram of sample collection points; (**B-C**) Habitat; (**D**) Ascomata; (**E**) Ascospores; (**F**) Mycelia; (**G**) Micromorphology of mycelia. (**H**) Phylogenetic tree of *Morchella spongiola* and 4 other fungal species based on Bayesian analysis of ITS gene sequences, with nodes annotated if they were supported by ≥ 0.60 Bayesian posterior probability. * Sequences submitted by our team

### Morphological analyses and molecular identification

Macroanatomical features were observed and documented in detail from fresh ascocarps in various developmental stages, based on methods described in Loizides et al. [25]. Pure culture isolations were obtained in potato dextrose agar (PDA) medium, from both ascospores and sterile ascocarp tissue of specimen M12-10. Macro- and micromorphological features were observed from the spore-isolated strain, which was inoculated on PDA and incubated at 25 °C, in both dark and daylight conditions. The terminology of the mycelium micromorphological features follows Qiao [26]. The internal transcribed spacer region of the nuclear rDNA locus (ITS), nuclear large subunit (nrLSU), the largest and second-largest subunits of RNA polymerase II (*RPB*1 and *RPB*2, respectively), and translation elongation factor 1 alpha (*TEF*1) were amplified by polymerase chain reaction (PCR). Phylogenetic analyses based on methods described in Meng et al. [27].

RETRACTED

### Genome assembly and assessment

Vegetative mycelia of M12-10 were cultivated in PDA medium in the dark at 25 °C for 5 days and then collected for genome sequencing. For genome sequencing, genomic DNA was extracted using a modified cetrimonium bromide (CTAB) procedure. Libraries for single-molecule real-time (SMRT) sequencing were constructed with an insert size of 20 kb using the SMRTbell Template Prep kit 1.0 (Pacific Biosciences, Menlo Park, CA, USA). Subsequently, the genome of M12-10 was sequenced using the PacBio Sequel platform using single-molecule real-time (SMRT) technology and Illumina NovaSeq PE150 from Genedenovo Biotechnology Co., Ltd (Guangzhou, China).

For genome assembly, the clean reads were corrected and assembled with the MECAT. To evaluate the completeness of the assembled genome, a Benchmarking Universal Single-Copy Orthologs (BUSCO) analysis was conducted using BUSCO v2.0 to search the assembled genome against the fungi_odb9 database, which comprises 290 cores conserved orthologs in total.

### Genome annotation

Genome component prediction included the prediction of coding genes, repetitive sequences, and noncoding RNAs. The available steps proceeded as follows: the Augustus 2.7 program was employed to retrieve the related coding genes; the interspersed repetitive sequences were predicted using RepeatMasker; the tandem repeats were analyzed using TRF (tandem repeats finder); transfer RNA (tRNA) genes were predicted with tRNAscan-SE; ribosomal RNA (rRNA) genes were analyzed using RNAmmer; and sRNA, snRNA, and miRNA genes were predicted via BLAST against the Rfam database [28].

We used three databases to predict gene functions: GO (Gene Ontology), KEGG (Kyoto Encyclopedia of Genes and Genomes), KOG (Clusters of Orthologous Groups) [29]. Meanwhile, biosynthetic gene clusters such as terpene synthases, nonribosomal peptide synthetases (NRPSs), and polyketide synthases (PKSs) in the *M. spongiola* M12-10 genome were identified via antiSMASH v5.0 [30].

### Comparative genomic analysis

All-vs-all BLASTP searches (with an E value cutoff of 10 − 5) were performed to identify paralogous or orthologous gene pairs, and query cov 30% were considered to be interspecies homologs according to the results of Diamond matching. Orthologous genes were clustered using OrthoMCL. To understand how gene families differ among species, a Venn diagram analysis was performed on the basis of the gene family number information to understand the common or unique genes between species. The upper number in each section represents the number of gene families, and the lower number represents the number of genes. BLASTN was used to identify synteny among the *Elata* clade phylospecies *M. importuna*/*Mel*-10 and *M. spongiola* M12-10, with the following parameters for genome-wide collinearity analyses: -evalue 1^e–5^ -perc_identity 80. To identify the synteny relationships between three *Esculenta* clades phylospecies *M. spongiola* M12-10, *M. parva*/*Mes*-7, and *M. vulgaris*/*Mes*-5, the longest coding DNA sequences (CDS) for each gene were identified in these three morels species based on MCscan. ClusterProfile v3.14.0 was used to conduct a GO and KEGG enrichment analysis with unique *M. spongiola* genes. For each species genome, Diamond was used in conjunction with OrthoMCL to identify homologous genes across species.

RETRACTED

The genus *Morchella* subgenome A was used to conduct a comparative genomic analysis. Gene families in *M. spongiola* M12-10 and 32 morels species (Table S1) were identified using OrthoFinder v2.5.151. Multiple sequence alignments of 182 single-copy homologous genes were performed using MAFFT v7.20552. We subsequently reconstructed the relationships of *Morchella* and related taxa on PhyloSuite v1.2.2. We used MrBayes v3.2.6 for BI phylogenetic analyses and ModelFinder to generate the best model. The uncorrelated lognormal relaxed molecular clock and the Yule speciation prior set were used to estimate the divergence time and the corresponding credibility intervals via BEAUti. Divergence times were estimated using MCMCTREE in BEAST 1, and secondary calibration points were obtained from BEAUti: Ascomycota/Basidiomycota (467.24-666.82 Mya), *Morchella*/*Verpa* (213.96-347.77 Mya), *Rufobrunnea* clades/*Morchella* (121.79-194.71 Mya), *Esculenta* clades/*Elata* clades (98.74-152.95 Mya), *Esculenta* clades (49.19–93.03 Mya), and *Elata* clades (70.49-109.89 Mya) [9, 10]. The Markov chain Monte Carlo (MCMC) analysis was set to 100 million generations, with sampling parameters for every 1000 generations. After discarding the first 10,000 (10%) trees as burn-in, the samples were summarized in a maximum clade credibility tree in TreeAnnotator v2.6.6 using a PP limit of 0.50 and summarizing the mean node heights. The means and 95% higher posterior densities (HPDs) of the age estimates were obtained from the combined outputs using Tracer. FigTree v1.4.2 and iTOL (https://itol.embl.de/) were used to visualize the resulting tree and to obtain the means and 95% HPD. A 95% HPD marks the shortest interval that contains 95% of the values sampled [31].

RETRACTED

## Results

### Strain isolation, identification, and redescription

Every year at the beginning of May, we collected wild morel near the Baokou River in the Qilian Mountains of Qinghai Province (Fig. 1A). Habitat: Near riverbeds, beaches, and sandy beaches, on soil under mixed forests dominated by *Populus przewalskii* Maxim., *Salix babylonica*, *Hippophae rhamnoides* L., *Rosa xanthina Lindl*, *Poa crymophila* cv. Qinghai, *Poa pratensis* L. cv. Qinghai (Fig. 1B-C).

Macroanatomical features description: Ascomata 22–45 mm high. Pileus 20–40 mm high × 10–15 mm wide; conical to bluntly conical; pitted and ridged. Ridges glabrous or finely tomentose; pallid to hazel when young, becoming dark grayish at maturity. Pits primarily vertically elongated; glabrous; brownish to yellowish tan. Stipe 20–25 mm high; 10–15 mm wide; more or less equal or sometimes basally (Fig. 1D). Micromorphological description: Ascospores (9.78–) 13.57–18.62 (–23.54) × (4.87–) 7.21–10.40 (–10.90) µm, Me = 15.74 × 8.57 μm, Qm = 1.83 (*n* = 50); elliptical; with irregular longitudinal and interconnecting transverse ridges; contents homogeneous; 8-spored; cylindrical; hyaline (Fig. 1E). The *Morchella spongiola* strain M12-10 was isolated from a typical *M. spongiola* fruiting body. Using a light microscope, the hyphae of M12-10 were hyaline (d = 15.01 ± 2.65 μm, *n* = 100), septate, and branching, and the clamp connections of hyphae were observed clearly, with no spores (Fig. 1F-G). The ITS sequence obtained with primers ITS1 and ITS4 was used to determine the identity in a BLAST nucleotide search of NCBI and exactly matched the ITS region of *Morchella spongiola* with 98% similarity. The search results indicated that strain M12-10 was a pure culture strain of *M. spongiola* (Fig. 1H). GenBank: ITS = MK937635; nrLSU = MW692181; *TEF*1 = OR351230; *RPB*1 = OR351231; *RPB*2 = OR351232.

### Characteristics of the *Morchella spongiola* genome

Third-generation-long fragment sequencing and two-mate-pair Illmuina jumping sequencing were used to de novo assemble the genomes of *M. spongiola* M12-10; we obtained 396,318 raw reads and 6132.9 million bases. The genome sequence was 51.7 Mb with a maximum sequence length of 4.09 Mb (Table 1); it consisted of 34 contigs with an N_50_ of 1.81 Mb and a GC content of 47.44% (Fig. 2). The final de novo genomic assembly results were submitted to NCBI, with the public accession number SRR18443859 (BioSample: SAMN26880165; BioProject: PRJNA781342). For genome composition, 9775 coding genes, 298 tRNA genes (Fig. 2 hollow circles), 43 rRNA genes (Fig. 2 hollow squares), 16 miRNA genes (Fig. 2 solid circles), and 18 snRNA (Fig. 2 hollow triangle) genes were predicted. The total number of DNA and RNA transposon elements (TEs) was 2177, with a length of 14,161,838 bp, accounting for 27.39% of the genome size. A total of 20 DNA TEs were detected, mainly Helitron and MITE, with numbers of 359 and 146, accounting for 13.97% and 1.32% of the length of the TEs, respectively. Gypsy (LTR) and L1 (LINE) were the main RNA TEs, with numbers of 550 and 80, covering 10.34% and 0.16% of the length of the TEs, respectively (Table 2). Overall, 1642 out of 1705 (96.31%) complete genes were identified using BUSCO with a 0.64% duplicate ratio represented in the assembled genome. Together, these results indicate that the *M. spongiola* M12-10 genome data were of high quality and sufficient for subsequent analyses.

RETRACTED

**Table 1:** The contig statistics of the assembled genome of *M. spongiola* M12-10

Parameter	M.spongiola M12-10
Scaffold characteristics	
Total number	34
Total length (bp)	51,704,070
Max length (bp)	19,119
N50 (bp)	1,814,099
N90 (bp)	1,000,758
G + C content (%)	47.44%
Genome characteristics	
Number of protein-coding genes	9775
Gene total length (bp)	13,321,592
Gene average length (bp)	1362.82
Gene/Genome (%)	2.57
Intergenic region length (bp)	38,383,478
GC content in intergenic region (%)	52.21%
Intergenic length/Genome (%)	72.42
BUSCOs	97.93%
Genomic annotation analysis	
KEGG annotation number genes	3234
KOG annotation number genes	6993
GO annotation number genes	3914
SwissPort annotation number genes	4580
Secondary metabolite biosynthesis gene clusters	9

**Fig. 2:** Circos plot of the *M. spongiola* M12-10 genome assembly. From the exterior to the interior, they are Chromosome (1–34), Repeat sequence density distribution (red), gene density distribution (blue), tRNA (hollow circles), rRNA (hollow squares), snRNA (hollow triangle), miRNA (solid circles), covariate linkage (number alignment results > 10 kb), respectively

**Table 2:** Statistics of repeat sequences in the *M. spongiola* M12-10 genome

Class	Order	Superfamily	Members	Length	% of genome
DNA transposons	TIR	CMC	84	36,242	0.07%
	TIR	MULE	47	8926	0.02%
	TIR	PIF	49	17,206	0.03%
	TIR	PiggyBac	7	3549	0.01%
	TIR	TcMar	78	131,817	0.25%
	TIR	hAT	99	15,883	0.03%
	Helitron	Helitron	359	7,220,598	13.97%
	Maverick	Maverick	19	5553	0.01%
	MITE	MITE	146	684,089	1.32%
	Unknow	Unknow	1	6284	0.01%
retrotransposons	LTR	P	11	926	0.00%
	LTR	Caulimovirus	1	58	0.00%
	LTR	Copia	176	22,206	0.04%
	LTR	ERV1	70	184,148	0.36%
	LTR	ERVK	40	167,346	0.32%
	LTR	Gypsy	550	5,347,943	10.34%
	LTR	Unknow	18	3690	0.01%
	LTR	Pao	71	8458	0.02%
	LINE	Jockey	17	25,578	0.05%
	LINE	L1	80	81,003	0.16%
	LINE	L2	31	38,958	0.08%
	LINE	R1	20	17,306	0.03%
	DIRS	I	11	69,617	0.13%
	DIRS	Ngaro	9	2897	0.01%
	SINE	Alu	7	3585	0.01%
Simple repeat	Simple repeat	Simple repeat	1	17,244	0.03%
Total	-	-	2177	14,161,838	27.39%

RETRACTED

### Functional annotations of *Morchella spongiola* genes

The results of the genome functional annotation are summarized in Table 1. All 9775 predicted genes were annotated in multiple public databases. A total of 7535 genes had homology to genes in at least one database, accounting for approximately 77.08% of the predicted genes.

In the GO classification analysis, the top five categories were cellular process, metabolic process, cell-cell part, catalytic activity, and organelle (Fig. 3A). In the KEGG pathway annotation results showed that 745, 296, 207, and 108 genes were enriched in the pathways of metabolic process, biosynthesis of secondary metabolites, biosynthesis of amino acids, and biosynthesis of antibiotics, respectively (Fig. 3B). Among the KOG categories, the number of genes related to posttranslational modification, protein turnover, chaperones (O), signal transduction mechanisms (T), RNA processing and modification (A), and intracellular trafficking, secretion, and vesicular transport (U) was greater than that of the other function-related genes (Fig. 3C). Antismash results from predicted genes found that the *M. spongiola* M12-10 genome had nine secondary metabolite clusters, which were rich in Nrps-like (nonribosomal peptide synthetase-like fragment) (33%), t1PKS (polyketides type 1) (11%), terpene (22%), indole (11%), NRP-metallophore (nonribosomal peptide metallophores) (11%), and fungal-RiPP (fungal RiPP with POP or UstH peptidase types and a modification) (11%) (Fig. 3D).

**Fig. 3:** Gene function annotation of the *M. spongiola* M12-10 genome. (**A**) GO enrichment analysis of annotated genes in M12-10. (**B**) KEGG pathway annotation of the genome of M12-10. (**C**) KOG function classification of annotated genes in M12-10. (**D**) Number and distribution of secondary metabolite gene clusters in the M12-10 genome

### Comparative genomic analysis

We conducted a comparative genomic analysis of the *M. spongiola* M12-10 genome against 32 other *Morchella* species. The genome size of the *M. spongiola* M12-10 genome was similar to that of the other *Esculenta* clade phylospecies *M. dunensis*/*Mes*-17 (Fig. 4A). The results showed that 266 essential families containing 21,678 genes were shared by 33 taxa, followed by 825 families containing 19,550 genes that were shared by 12 *Esculenta* clades, and 576 families containing 19,550 genes that were shared by 19 *Elata* clades; there were 24, 140, and 877 species-specific families containing 30, 925, and 140 genes in the three classifications, respectively (Fig. 4B-D). Notably, 925 unique genes in *M. spongiola* M12-10 were analyzed using multiple functional databases. Functional analysis showed that two unique genes encoded proteins related to molecular function regulation, transcription factor activity, and protein binding (Fig. 4E, F). GO enrichment analysis revealed that the unique *M. spongiola* M12-10 genes were significantly enriched in the following terms: biological regulation, response to stimulus, signaling, growth, reproduction, and reproductive process, and two unique genes encoded proteins related to molecular function regulation, transcription factor activity, and protein binding (Fig. 4E). KEGG analysis revealed that these unique genes were enriched in several pathways: starch and sucrose metabolism, carbon metabolism, amino acid metabolism, and glycan biosynthesis and metabolism. Most genes that were only present in *M. spongiola* M12-10 were significantly enriched in signal transduction, such as the phosphatidylinositol signaling system (Fig. 4F).

RETRACTED

**Fig. 4:** Genome comparison analysis between *M. spongiola* M12-10 and 32 other *Morchella* phylospecies. (**A**) Genome assembly size of 33 *Morchella* phylospecies. (**B-D**) Petal diagram of the gene families in 33 species. The middle circle is the number of gene families shared by all species, and the number of unique gene families is on the side. (**E**) GO terms of *M. spongiola* M12-10. A total of 21,678 genes (gray) and 925 unique genes (blue) were functionally interpreted. (**F**) KEGG classification analysis of *M. spongiola* M12-10

The genomic collinearity analysis showed that several chromosomal segments in the *M. importuna*/*Mel*-10 genomes were condensed into one segment in *M. spongiola* M12-10, with some inversions (Fig. 5A). Some orthologs in *M. spongiola* M12-10 had many-to-one relationships. At least two query genes in *M. spongiola* M12-10 matched the same ortholog in the reference species. Notably, significant genomic regions of *M. spongiola* M12-10 could not be collinearly coupled with those in the *Morchella* genome, supported by a 23.59% with *M. importuna*/*Mel*-10 collinearity rate (the ratio of colinear ortholog pairs to all ortholog pairs), which was less than that between M12-10 and *M. vulgaris*/*Mes*-5 (94.61%), and *M. prava*/*Mes*-7 (95.30%), the results indicated that *M. spongiola* M12-10 is phylogenetically distant from those three morel species (Fig. 5B). In addition, despite the high degree of collinearity of most scaffolds, the genomes of M12-10 and *M. vulgaris*/*Mes*-5 had undergone some complex interchromosomal rearrangements. Similar rearrangements also occurred comparing M12-10 and *M. prava*/*Mes*-7 chromosomes, which may suggest that chromosome rearrangement in *M. spongiola* M12-10 during evolution. However, this phenomenon could also be caused by the low quality of *M. spongiola* M12-10 genome sequence data.

RETRACTED

**Fig. 5:** Dual synteny plot showing genome collinearity. (**A**) Different colored lines were used to connect the orthologous pairs between *M. spongiola* M12-10 and *M. importuna*/*Mel*-10; (**B**) Syntenic analysis via comparisons the longest CDS of *M. spongiola* M12-10 with *M. parva*, *M. spongiola* M12-10 with *M. vulgaris*. The values on the right are collinearity rate. Fruiting bodies of *Morchella* species downloaded from Mycocosm Portals (doe.gov)

### Phylogenetic analysis and evolution of the Genus *Morchella*

A phylogenetic and time-calibrated phylogenetic tree was constructed using 182 single-copy orthologs from 33 *Morchella* phylospecies, and the topology of the tree was consistent with our current understanding of the relationships among these taxa (Fig. 6). The phylogenetic analysis indicated that *M. spongiola* M12-10 is a distinct species, similar in age to the *Esculenta*-like stature phyolspecies *M. parva*/*Mes*-7. The divergence time of the genus *Morchella* was approximately to be 274.04 million years ago (Mya) (HPD% 272.03–275.96). The *Morchella* species diverged into three clades; the first clade diverged an estimated 154.06 Mya (*Rufobrunnea* clade, 95% HPD 152.14-156.02), closely related to the Triassic junction; the second clade diverged an estimated 101.9 Mya (*Esculenta* and *Elata* clades, 95% HPD 87.25–115.00), closely related to the Late Cretaceous junction; the *Esculenta* clades diverged 73.77 Mya (95% HPD 65.03–103.87) and the *Elata* clades diverged 84.54 Mya (95% HPD 50.58–97.42). *M. spongiola* M12-10 was allied with another *Esculenta* clade, *M. parva*/*Mes*-7, both of which are older species that were separated by approximately 12.85 Mya (95% HPD 0.25–17.45), when the Qinghai-Tibet Plateau experienced the first historical geological uplift.

**Fig. 6:** Phylogenetic chronogram showing the evolutionary dating time of the genus *Morchella* using 33 phylospecies. The tree was estimated using Bayesian analysis of 182 single-copy orthologous genes in the MCMC tree. Fruiting bodies of *Morchella* species downloaded from Mycocosm Portals (doe.gov)

## Discussion

### *Morchella spongiola* genome

In this study, we generated a representative assembly for a high-quality *Morchella spongiola* M12-10 draft genome. The 1k genome projects and other researchers have sequenced 35 *Morchella* species, all of which have been released on the JGI website, playing a significant role in promoting related scientific research [25]. The genome of *M. spongiola* M12-10 detailed in this paper is the first reported genome of this species. Generally, *M. spongiola* is slightly larger than *M. septentrionalis* (51.47 Mb), *M. dunensis* (51.33 Mb), and *M. esculenta* (51.15 Mb) in genome size. The sizes were different in the Gypsy (LTR) and Tad1 (LINE) analyses, with numbers of 550 and 214, covering 10.34% and 33.00% of the length of the TEs of *M. spongiola*, in contrast to 29.30% and 3.73% for *M. crassipes*, respectively. A total of 9775 genes were annotated in the *M. spongiola* M12-10 genome, which is slightly different from the number of genes annotated in the genomes of *M. crassipes* (11,565 genes), *M. sextelata* (9550 genes), and *M. importuna* (16,099 genes). This genome sequence will aid germplasm management, molecular breeding, and pharmaceutical and ecological studies on plants in this family. *M. spongiola* M12-10 is one of the most highly priced edible mushrooms and a rich source of bioactive substances, with numerous beneficial medicinal properties, such as biologically active polysaccharides, polyphenols, protein hydrolysates, γ-aminobutyric acid, sterols, flavonoids, furan compounds, mushroom alcohols, volatile substances, and tocopherols [32–37]. Previously, a platelet colony inhibitor with potency 2–3 times higher than that of aspirin and a melanogenesis inhibitor that inhibits tyrosinase were isolated from the fermentation broth of *Morchella*, but the key roles of the biologically active substances are not clear [38–41]. In the genome of *M. spongiola* M12-10, we detected multiple clusters of secondary metabolite genes, such as terpene, indole, fungal-RiPP, which means that there is potential antioxidant activity. Additional studies are needed to clarify the functions of these candidate genes and the molecular mechanisms of biologically active substances.

RETRACTED

### Phylogenetic analysis

Phylogenetic analysis indicated that the *M. spongiola* M12-10 and *M. parva* form a monophyletic branch. Surprisingly, the name *M. spongiola* was described by Richard et al. [11] to be a later synonym of the well-established and epityfied taxon *M. vulgaris*, whereas *M. parva* also probably corresponds to what has been labeled ‘‘*M. vulgaris*’’. However, there are significant morphological variations in the hymenophore (Fig. 5B). *M. spongiola* is primarily distributed in forests containing *Ulmaceae* Mirb., *Populus tomentosa* Carr, and *Hippophae rhamnoides* L., with occasional occurrences alongside herbaceous plants and sporadically with other plant species. *M. spongiola* can typically be recognized by its sponge-like appearance, contorted, asymmetrical, and highly irregular pits, as well as bluntly rounded ridges that tend to darken as the fungus matures. In contrast, the micromorphological ascospores of *M. spongiola* strain M12-10 measure (9.78-) 13.57–18.62 (-23.54) × (4.87-) 7.21–10.40 (-10.90) µm, while those of *M. prava* range from (16-) 17–21 (-24) x (8-) 10–12 (-13) µ [44], indicating a notable difference in spore size between the two species. Specifically, *M. vulgaris* seems to have a more restricted distribution and is currently considered narrowly endemic from Europe to India and China, primarily associating with poplar and pine trees [42]. *M. prava*, a species commonly found within the latitudes of 43–50°N in North America, can be distinguished by its esculenta-like appearance, characterized by a twisted stature, contorted pits, and asymmetrical or irregular ridges [43, 44]. Therefore, these mixed features are considered significant enough to propose a difference among the three species. Most *Morchella* species appear to exhibit continental endemism, provincialism, and cryptic speciation, which has greatly facilitated the reconstruction of their historical biogeography. It is only through the use of multilocus analyses, such as population genetics, morphological, developmental, and behavioral analyses, chemotaxonomy, cytology, ultrastructural and reproductive studies, integrative approaches, and careful evaluations of all lines of evidence that a number of closely related and insufficiently clarified lineages in *Morchella* have been identified [10].

### The historical biogeography of *M. spongiola* in QTPs

Divergence time estimation showed that *M. spongiola* M12-10 and *M. parva* diverged from a recent common ancestor at approximately 12.85 Mya (in the Miocene epoch), while *M. vulgaris* and *M. parva*-*M. spongiola* M12-10 diverged approximately 16.13 Mya (Late Oligocene). Previously, it is speculated that *Morchella* originated in western North America during the Late Jurassic period and diverged into the basal lineage *M. rufobrunnea* [11, 45, 46]. A further study by Loizides et al. [25] revealing that the origin of the two *Rufobrunnea* clade phylospecies, *M. anatolica*, and *M. rufobrunnea*, is Mediterranean rather than North American or Asian. In our study, *M. anatolica* and *M. rufobrunnea* are also the earliest-diverging lineages and the speciation of *M. spongiloa* is strongly linked to the first uplift event of the QTPs. Tectonic activity and climate change during geological periods can not only create barriers to geographic isolation that contribute to species differentiation and diversity but can also expand species ranges and increase biological exchange between regions by reducing barriers to biological dispersal [47–49]. We therefore presume that the *M. vulgaris* was closer ancestor species of *M. spongiola* and *M. parva*, and the paleogeological changes of QTPs were most likely the key factors responsible for the diverging and diversifying morphological appearance of the *Morchella spongiola*.

RETRACTED

## Conclusions

The high-quality genome assembly of *Morchella spongiola* M12-10 from the Qinghai-Tibet Plateau and the comparative genomic analysis with 32 other *Morchella* species indicated unique features in its genome size and genomic components. Our results clarified that *M. spongiola* is a distinct phylospecies rather than a synonym of *M. vulgaris* based on morphological, molecular biological, genomic, and comparative genomic analyses. Meanwhile, the formation and evolutionary processes of *M. spongiola* M12-10 on the QTPs are strongly influenced by the tectonic uplift and geological movements of the plateau. The new genomic data described here lay the foundations for future studies to clarify the mechanisms of the special biological characteristics of *M. spongiola*, as well as for future comparative genomic and genetic studies across different fungal lineages.

### Electronic supplementary material

Below is the link to the electronic supplementary material.

Supplementary Material 1

## Data Availability

All data generated or analyzed during this study are included in this published article and the complete chromosome genome sequences of *M. spongiola* M12-10 are deposited in the Genbank accession number SRR18443859, BioSample: SAMN26880165, BioProject: PRJNA781342, respectively. GenBank accession number of *M. spongiola* M12-10 in five genes (rDNA): ITS = MK937635; nrLSU = MW692181; *TEF*1 = OR351230; *RPB*1 = OR351231; *RPB*2 = OR351232.

## Abbreviations

QTPs: Qinghai-Tibet Plateau subkingdoms
Mya: million years ago
JGI: joint genome institute
SMRT: single molecule real time
ITS: internal transcribed spacer
nrLSU: nuclear large subunit
*RPB*1: largest subunits of RNA polymerase I
*RPB*2: second-largest subunits of RNA polymerase II
*TEF*1: translation elongation factor 1 alpha
PCR: polymerase chain reaction
NCBI: National Center for Biotechnology Information
BLAST: Basic Local Alignment Search Tool
TEs: transposon elements
LTR: long terminal repeat-retrotransposons
LINE: long interspersed nuclear elements
BUSCO: Benchmarking Universal Single-Copy Orthologs
GO: Gene Ontology
KEGG: Kyoto Encyclopedia of Genes and Genomes
KOG: Clusters of Orthologous Groups
rRNA: Ribosomal RNA genes
tRNA: transfer RNAs genes
SSRs: simple sequence repeats
PCR: polymerase chain reaction
BI: Bayesian Inference
Nrps-like: nonribosomal peptide synthetase-like fragment
t1PKS: polyketides type 1
NRP-metallophore: nonribosomal peptide metallophores
fungal-RiPP: fungal RiPP with POP or UstH peptidase types and a modification
GCPSR: genealogical concordance phylogenetic species recognition
